# Artificial Intelligence in Modern Medicine – The Evolving Necessity of the Present and Role in Transforming the Future of Medical Care

**DOI:** 10.7759/cureus.8041

**Published:** 2020-05-09

**Authors:** Pradnya Brijmohan Bhattad, Vinay Jain

**Affiliations:** 1 Internal Medicine, East Tennessee State University, Johnson City, USA; 2 Radiology, James H. Quillen Veterans Affairs Medical Center, Johnson City, USA

**Keywords:** artificial intelligence, digital twin, machine learning

## Abstract

The dexterity of computer systems to resemble and mimic human intelligence is artificial intelligence. Artificial intelligence has reformed the diagnostic and therapeutic precision and competence in various fields of medicine. Artificial intelligence appears to play a bright role in medical diagnosis. Computer systems using artificial intelligence help in the assessment of medical images and enormous data. This research aims to identify how artificial intelligence-based technology is reforming the art of medicine. Artificial intelligence empowers providers in improving efficiency and overall healthcare. Newer machine learning techniques lead the automatic diagnostic systems. Areas of medicine such as medical imaging, automated clinical decision-making support have made significant advances with respect to artificial intelligence technology. With improved diagnosis and prognosis, artificial intelligence possesses the capability to revolutionize various fields of medicine. Artificial intelligence has its own limitations and cannot replace a bedside clinician. In the evolving modern medical digital world, physicians need to support artificial intelligence rather than fear it replacing trained physicians for improved healthcare.

## Introduction and background

Artificial intelligence involves the use of mathematical computational techniques with developing algorithms that mimic human intelligence [1]. A study database that focuses on the question is created; this data can be from diverse sources such as wearable devices to electronic medical records. Artificial intelligence mathematical models suitable for problem-solving are identified and then implemented by way of a programming language. Algorithms are used to obtain results/answers to the initial question and these results are further analyzed [1-4]. The emerging newer technology with advances in machine learning is transforming medical care [2,5].

## Review

Artificial intelligence - What is it?

Artificial intelligence (AI) is the driving force of the latest technological developments in medical diagnosis with a revolutionary impact [2,4]. Artificial intelligence can enhance productivity. AI mainly augments human intelligence due to its ability to automatize certain tasks [6,7].

Association for Computing Machinery (ACM) computing classification scheme categorizes artificial intelligence technology in three classes:

1. AI techniques - advanced mathematical models, for instance, machine learning, expert systems that allow performing tasks that are usually done by humans. Refer to Table 1* *below.

2. AI functional applications - computer vision and such functions can be understood by different AI techniques. Refer to Table 2 below.

3. AI application fields - diverse disciplines where AI techniques/functional applications may play a promising role such as in medical sciences in the fields of medical imaging, public health, genetics, drug discovery, medical informatics [3-5, 8].

**Table 1:** Artificial intelligence techniques Refs. [1, 3-5]

Artificial intelligence techniques
A. Machine learning: supervised learning, unsupervised learning, reinforced learning, multitask learning, rule learning, deep learning, latent representation, logical and relational learning, instance-based learning, probabilistic graphical models, bio-inspired approaches, classification and regression trees, support vector machines, neural networks
B. Logic programming: expert systems, description logistics, logic programming general
C. Fuzzy logic
D. Ontology engineering
E. Probabilistic reasoning

**Table 2:** Artificial intelligence functional applications Refs. [1, 3-6]

Artificial intelligence functional applications
1. Computer vision: image and video segmentation, character recognition, object tracking, scene understanding, augmented reality, computer vision (general)
2. Control methods
3. Planning and scheduling
4. Robotics
5. Natural language processing
6. Distributed AI
7. Predictive analytics
8. Knowledge representation and reasoning
9. Speech processing

Machine learning, digital twins in healthcare

Digital twins can mirror real and may lead to early diagnosis. Digital technology links the real and virtual worlds by using artificial intelligence in order to transform data into real construction [9-12]. Digital twins allow formulating an individualized physiological model with a promising potential to assess the efficacy of tailored treatments and precision medicine. A digital twin has the potential to predict procedural outcomes, to help provide tailored treatment and individualized treatment plans [9-11].

Machine learning is a type of artificial intelligence wherein computers construct algorithms from data to learn [13]. Newer machine learning techniques lead the automatic diagnostic systems. Deep learning helps put together multilevel data such as images, text, sound. Smart data analysis is an important aspect of technological advancements in medicine [14,15]. Cardiac imaging such as echocardiography, cardiac magnetic resonance imaging have been some of the areas of testing artificial intelligence-based learning techniques in medicine [15-17].

What beholds for artificial intelligence in medical care

AI has the potential to further improve patient care due to its ability to interpret more detailed and comprehensive data and as such, AI in medicine should be welcomed [16,17]. Incorporating artificial intelligence in our clinics has the potential to enhance physician efficiency. AI does not have the potential to replace the physician's expertise in the clinical presentation which will remain the vital aspect of medical care [16,18]. Appropriate application of artificial intelligence models has a promising role in health maintenance and preventative programs if we can identify the areas where to apply these AI models. Artificial intelligence is already in medicine especially, the computer vision in medical imaging. Safety and precision of AI algorithms need to be well defined and further established before artificial intelligence is integrated into clinical practice [17,18,19].

In the ever-digitalizing world of medicine and its diverse branches, physicians need to enthusiastically support artificial intelligence rather than fear it replacing trained physicians. Physicians will need to learn on appropriate application and interpretation of artificial intelligence models in the new age of artificial intelligence. Artificial intelligence has its own limitations and cannot replace a bedside clinician [16,19].

The age of artificial intelligence has the potential to improve the practice of future medicine - making treatment and medical care more efficient, accurate, comprehensive and individualized [18-20].

## Conclusions

AI has the potential to reform medical care in the upcoming era. It has already proven to enhance efficiency in healthcare delivery. The use of AI techniques can interpret comprehensive data in a short period of time efficiently and accurately thereby enhancing patient care. AI has limitations and cannot replace the bedside clinical interpretation of a physician. AI is already here in the present times with the current medical practice, for instance, computer vision in medical imaging. The diverse universe of medicine is ever digitalizing with rapid technological advancements. The use of AI needs to be incorporated with regards to the application and interpretation of AI models in the appropriate clinical settings. The new age demands smart use of AI to transform medical care to make it even more efficient and accurate.

The use of telehealth clinics, remote monitoring of cardiac devices, interpreting imaging studies remotely by radiologists, and cardiologists on the electronic health records are all here and are widely being utilized in daily life especially in this Coronavirus Disease 2019 (COVID-19) era. The advent of medical conferences via online classes and social media is a new form of technological advancements in medical education. Thus, the use of AI is already on its way to make a better future in the post-COVID-19 pandemic era.
